RETRACTED

# COVID-19 and Living Donor Kidney Transplantation in Naples during the Pandemic

**DOI:** 10.1155/2020/5703963

**Published:** 2020-10-15

**Authors:** Gaia Peluso, Silvia Campanile, Alessandro Scotti, Vincenzo Tammaro, Akbar Jamshidi, Luigi Pelosio, Marcello Caggiano, Teresa Pagano, Francesco Cuozzo, Fabrizio D'Ambrosio, Armando Calogero, Concetta Dodaro, Caterina Sagnelli, Nicola Carlomagno, Michele L. Santangelo

**Affiliations:** ^1^Operative Unit (O.U.) of General Surgery and Kidney Transplantation-Advanced Biomedical Science Department, University Federico II of Naples, Via S. Pansini 5 -80131 Naples, Italy; ^2^Department Mental Health and Public Medicine, Section of Infectious Diseases, University of Campania Luigi Vanvitelli, Naples, Italy

## Abstract

**Introduction:**

SARS-CoV-2 is a virus that causes a potentially deadly syndrome that affects especially the respiratory tract. Kidney-transplanted patients are immunosuppressed and more susceptible to viral infections. We have examined our transplantation activity to explore the future role of kidney transplantation from deceased and living donors in COVID-19 era. *Patients and Methods*. The activity of our transplant center of Naples (one of the two transplant centers in Campania, South Italy) continued during the COVID-19 pandemic. We have analysed the kidney transplants carried out between March 9 and June 9, 2020, comparing these data with the numbers of procedures performed in the two previous years. Moreover, we have considered the possibility of performing living donor transplants during a worldwide pandemic.

**Results:**

From March 9, 2020, when the Italian lockdown begun, till June 9, 2020, five kidney transplants have been performed at our transplant center in Naples, all from deceased donors. The donors and the recipients have been screened for COVID-19 infection, and the patients, all asymptomatic, followed strict preventive measures and were fully informed about the risks of surgery and immunosuppression during a pandemic. All the transplanted patients remained COVID negative during the follow-up. The number of transplants performed has been constant compared to the same months of 2018 and 2019. In agreement with the patients, we decided to postpone living donor transplants to a period of greater control of the SARS-CoV-2 spread in Italy.

**Conclusion:**

Deceased donor kidney transplantation should continue, especially in a region with moderate risk, like Campania, with a more careful selection of donors and recipients, preferring standard donors and recipients without severe comorbidities. Living donor transplantation program, instead, should be postponed to a period of greater control of the SARS-CoV-2 spread, as it is an elective surgery and its delay does not determine additional risks for patients.

RETRACTED

## 1. Introduction

SARS-CoV-2 is a single-stranded and positive-sense RNA virus, belonging to the Coronaviridae family that causes a flu-like syndrome, potentially deadly. It mainly involves the respiratory tract and can manifest itself with symptoms of varying intensity (e.g. fever, cough, dyspnoea to tracheitis-bronchitis, and pneumonia). The interest of the digestive tract is also characteristic [1].

In Italy, the first two cases, two Chinese citizens, have been reported in Rome on January 30, 2020, and since then, the infection has spread to include to date on June 15, 2020, 237.290 patients, with more than 34.000 deaths [2, 3]. From March 9, 2020, the Italian government has established several measures to obtain social distancing and ordered a country-wide lockdown.

Kidney-transplanted patients, because of immunosuppression after transplantation, are a more susceptible population to viral infections and pneumonia. Solid information about epidemiology, clinic, and management of SARS-CoV-2 infections in kidney transplant recipients are still few and unclear [4].

A recent Italian survey and consensus has tried to fill some gaps about this disease in transplanted patients. The authors have highlighted a decrease of the transplantation activities, especially for living donor transplants, and have presented some recommendation [5].

We have explored the transplantation activity of our transplant center in a region, the Campania, which has more than 6 million inhabitants and a moderate risk for COVID-19 infection, with the aim to establish the future objectives, focusing on the role of living donation during the pandemic.

## 2. Patients and Methods

In Campania, a region in South Italy, there are two kidney transplant centers, ours in Naples and the other one in Salerno, each with more than 250 patients on the waiting list for kidney transplant from deceased donors. The living donor kidney transplants are, instead, performed only by our center, and as of March 9, 2020, we were studying 10 potential donor/recipient couples. The activity of our transplant center of Naples continued during the COVID-19 pandemic. We have analysed the number of kidney transplants performed since the beginning of Italian lockdown, on March 9, 2020, till June 9, 2020. Then, we have compared these data with the numbers of procedures carried out in the same three months in the previous two years. Moreover, we have considered the feasibility to execute living donor transplant during a worldwide pandemic, taking into consideration the couples of patients we are following for this procedure.

RETRACTED

## 3. Results

In the three months, between March 9, 2020, when the Italian lockdown begun, and June 9, 2020, five kidney transplants have been performed at our transplant center in Naples, all from deceased donors. The kidneys came from standard donors, deceased for head injury or brain haemorrhage, who underwent nasopharyngeal swab at the time of hospitalization and bronchoalveolar lavage before donation, as established by national directives. The recipients had strictly adhered to the protective measures imposed by the Italian government and received by our hospital and had not had any contact with suspicious people or stayed in high risk areas; but most of all, they did not show any symptoms suggestive of COVID-19 infection and have been screened at the time of hospitalization with a nasopharyngeal swab and serological exams. The patients were 4 males and 1 female, all younger than 60 years old. They have been all fully informed about the benefits and the risks associated with kidney transplantation and about the risks of starting an immunosuppressive treatment during a pandemic. Moreover, they accepted the hazards related to structural changes made to the ward and the operating room usually used for transplantation, due to the COVID-19 emergency. The surgical procedures have been executed without complications, and all the patients have been discharged with a valid kidney function and without suspicious symptoms. The immunosuppressive therapy was our standard treatment and consisted in Basiliximab, at induction and on the 4th postoperative day, corticosteroids in decreasing doses, and Tacrolimus. During the follow-up, the patients are still asymptomatic and have been tested with serological tests that resulted negative for anti-SARS-CoV-2 antibodies.

None of these transplants, however, have been performed in March, the month in which the spread of the virus begun. The first one has been carried out on April 9, 2020, when the protocols for the virus' detection and the protective measures had already been adopted.

The transplantation activity in our center has been constant if compared to the same three months in the previous two years, in which there has been a reduction in the number of donations in Campania. In 2018 and 2019, between March 9 and June 9, respectively, 6 transplants were performed each year in our center. The difference from previous years has been a smaller number of observations for donation and of marginal donors.

Regarding live donor transplantation, we have decided to delay the procedures in agreement with the patients, being transplants to be organized in election. The only doubt arose about our preemptive patient, whose benefit could be greater than the high risk posed by the COVID-19 pandemic. Even in this case, after long discussion with the donor and the recipient about the hazards and the advantages of transplantation and dialytic treatments, it was decided to postpone the transplantation until the end of the phase two of the containment process of the pandemic [6].

RETRACTED

## 4. Discussion

The lack of data regarding kidney transplantation during COVID-19 pandemic has made the transplantation activity difficult in recent months, representing a real challenge for surgeons and clinicians.

Infection is a common complication that arises after kidney transplantation, and the respiratory tract is one of the most frequently infected organs. The onset may be frequently early in the first postoperative months with unusual symptoms and rapid progression. Transplanted patients, usually, have a poorer prognosis compared to the general population, and moreover, molecular cross-reactivity after respiratory viral infection can determine an acute rejection in transplanted recipients [1].

The Italian survey has highlighted that most of transplant centers have drastically diminished their activity, especially in the areas where the incidence of COVID-19 infection was higher [5]. Our center is situated in a region with moderate risk, so we have decided to continue with our activity regarding deceased donor transplants, however making a more careful selection of donors and recipients. We have preferred standard donors and selected recipients without severe comorbidities, which could result in an increased risk of infection and death for COVID-19, as suggested by some authors [7–11]. During those months, we did not have any urgent patients on the waiting list, such as hyperimmune or patients with difficult vascular access; in these cases, the transplant could be life-saving and so we would have carried out the procedure even in the case of no standard donors. A careful screening of the patients was performed, and the staff that treated them has been reduced to a minimum and has been subjected to close monitoring. None of our patients has been infected by SARS-CoV-2 during hospitalization or follow-up, supporting the preliminary data that suggest a low risk of acquiring the viral infection by transplanted patients, with a clinical course not different from that of nontransplant individuals [4, 12–14]. However, the affected patients seem to have a higher risk of becoming seriously ill and have an increased rate of mortality, especially in older patients [11, 12, 15–18].

The immunosuppressive agents usually used to reduce the incidence of rejection of transplanted organs reduce also the immunological response of the patient, increasing its susceptibility to opportunistic infections [19]. All the data show the need to reduce the immunosuppression therapy in symptomatic and asymptomatic patients [5, 20–23]. As we did not have any infected patient at the moment, we have administered the usual immunosuppressive therapy, at the minimum effective doses [24].

RETRACTED

The kidneys from deceased donors should always be transplanted; otherwise, they would be lost, and therefore, we continued with the deceased donor transplants, even though we did not perform any transplant in March, because intensive cares were engaged in the COVID-19 emergency. On the other hand, we suspended the living donor transplantation program, as it is a planned surgery that may be postponed to a period of greater control of the SARS-CoV-2 virus spread without additional risks for patients. This decision was made in agreement with the patients, who found it safer to continue dialysis rather than undergo to a surgery procedure and to a long hospitalization in COVID-19 era. Even our only preemptive patient decided to delay the transplantation till the end of the lockdown, accepting the probability of starting dialysis treatment. The temporary suspension of elective living donor transplantation is supported by the most recent recommendations worldwide [5, 15, 25–27].

## 5. Conclusion

In conclusion, we support the idea to suspend the elective living donor kidney transplantation till the end of the COVID-19 pandemic so as to not create additional risks for healthy patients. However, we suggest continuing with deceased donor transplantation in areas with low or moderate risk of SARS-CoV-2 spread, adopting specific preventive measures and screening programs for donors, recipients, and medical staff.

## Data Availability

Data are available on request.

## References

[1] Ju C. R., Lian Q. Y., Zhang J. H. (2020). Recommended prophylactic and management strategies for severe acute respiratory syndrome coronavirus 2 infection in transplant recipients. *Chronic Diseases and Translational Medicine*.

[2] http://www.salute.gov.it/portale/nuovocoronavirus/dettaglioContenutiNuovoCoronavirus.jsp?area=nuovoCoronavirus&id=5351&lingua=italiano&menu=vuoto

[3] Remuzzi A., Remuzzi G. (2020). COVID-19 and Italy: what next?. *The Lancet*.

[4] Zhang H., Chen Y., Yuan Q. (2020). Identification of kidney transplant recipients with coronavirus disease 2019. *European Urology*.

[5] Vistoli F., on behalf of the Italian National Kidney Transplantation Network, Furian L. (2020). COVID-19 and kidney transplantation: an Italian survey and consensus. *Journal of Nephrology*.

RETRACTED

[6] http://www.governo.it/it/coronavirus-normativa

[7] De Rosa P., Santangelo M., Scala A. (2006). Difficult vascular conditions in kidney transplantation. *Transplantation Proceedings*.

[8] Bellini M. I., Tortorici F., Capogni M. (2020). Kidney transplantation and the lockdown effect. *Transplant International*.

[9] Incollingo P., Peluso G., Pelosio L. (2019). Ethical issues in the use of suboptimal kidneys for transplants: an Italian point of view. *Transplantation Proceedings*.

[10] De Rosa P., Santangelo M., Ferrara A. (2004). Suboptimal kidney: the experience of a single transplant unit. *Transplantation Proceedings*.

[11] Santangelo M., Zuccaro M., De Rosa P. (2007). Older kidneys donor transplantation: five years' experience without biopsy and using clinical laboratory and macroscopic anatomy evaluation. *Transplantation Proceedings*.

[12] Montagud-Marrahi E., Cofan F., Torregrosa J. V. (2020). Preliminary data on outcomes of SARS-CoV-2 infection in a Spanish single center cohort of kidney recipients. *American Journal of Transplantation*.

[13] Gandolfini I., Delsante M., Fiaccadori E. (2020). COVID-19 in kidney transplant recipients. *American Journal of Transplantation*.

[14] Piscitelli P., Santoriello A., Buonaguro F. M. (2009). Incidence of breast cancer in Italy: mastectomies and quadrantectomies from 2000 to 2005. *Journal of Experimental & Clinical Cancer Research*.

[15] Pascual J., Melilli E., Jiménez-Martín C. (2020). COVID-19–related mortality during the first 60 days after kidney transplantation. *European Urology*.

[16] Nacif L. S., Zanini L. Y., Waisberg D. R. (2020). COVID-19 in solid organ transplantation patients: a systematic review. *Clinics*.

[17] Akalin E., Azzi Y., Bartash R. (2020). COVID-19 and kidney transplantation. *New England Journal of Medicine*.

[18] Criscitiello C., Giuliano M., Curigliano G. (2015). Surgery of the primary tumor in de novo metastatic breast cancer: to do or not to do?. *European Journal of Surgical Oncology*.

[19] Fishman J. A. (2007). Infection in solid-organ transplant recipients. *New England Journal of Medicine*.

[20] Nair V., Jandovitz N., Hirsch J. S. (2020). COVID-19 in kidney transplant recipients. *American Journal of Transplantation*.

[21] Santangelo M. L., Criscitiello C., Renda A. (2015). Immunosuppression and multiple primary malignancies in kidney-transplanted patients: a single-institute study. *BioMed Research International*.

[22] Ritschl P. V., Nevermann N., Wiering L. (2020). Solid organ transplantation programs facing lack of empiric evidence in the COVID-19 pandemic: a By-proxy society recommendation consensus approach. *American Journal of Transplantation*.

RETRACTED

[23] Pisani A., Sabbatini M., Imbriaco M. (2016). Long-term effects of octreotide on liver volume in patients with polycystic kidney and liver disease. *Clinical Gastroenterology and Hepatology*.

[24] Peluso G., Incollingo P., Carlomagno N. (2019). Our timing to remove peritoneal catheter dialysis after kidney transplant. *Transplantation Proceedings*.

[25] Cacciola R. (2020). Response to "The COVID-19 outbreak in Italy: initial implications for organ transplantation programs". *American Journal of Transplantation : Official Journal of the American Society of Transplantation and the American Society of Transplant Surgeons.*.

[26] Creta M., Calogero A., Sagnelli C. (2019). Donor and recipient outcomes following robotic-assisted laparoscopic living donor nephrectomy: a systematic review. *BioMed Research International*.

[27] Ferrarese A., Pozzi G., Borghi F. (2016). Informed consent in robotic surgery: quality of information and patient perception. *Open Medicine*.

